# Incentive Nursing can Effectively Improve the ESCA Level of Patients with Endometrial Cancer after Laparoscopic Hysterectomy

**DOI:** 10.1155/2022/5159009

**Published:** 2022-07-12

**Authors:** Ju Zong, Liping Chen, Jie Chen

**Affiliations:** ^1^Department of Medical Oncology, The First Affiliated Hospital of Soochow University, Soochow, China; ^2^Department of Gynecology, The First Affiliated Hospital of Soochow University, Soochow, China

## Abstract

**Objective:**

To investigate the effect of incentive nursing on the rehabilitation of patients with endometrial cancer after laparoscopic hysterectomy.

**Methods:**

A total of 110 patients with endometrial cancer receiving laparoscopic hysterectomy in our hospital from October 2017 to July 2020 were recruited and assigned at a ratio of 1 : 1 to receive either routine nursing (control group) or incentive nursing plus routine care (study group). Outcome measures included the self-rating anxiety scale (SAS) score, Hamilton depression scale (HAMD) score, the exercise of self-care agency (ESCA) score, postoperative rehabilitation outcomes, the incidence of nursing complications, and nursing satisfaction.

**Results:**

Patients receiving incentive nursing showed significantly lower SAS scores and HAMD scores, and a higher ESCA score versus patients given routine care alone (*P* < 0.05). Incentive care resulted in a shorter length of hospital stay and postoperative time of out-of-bed activities and exercises versus routine care (*P* < 0.05). Incentive care was associated with a significantly lower incidence of nursing complications and higher nursing satisfaction versus routine nursing (*P* < 0.05).

**Conclusion:**

Incentive nursing can effectively improve the ESCA level of patients, promote postoperative recovery, and reduce the incidence of complications, so it is worthy of clinical promotion.

## 1. Introduction

Endometrial cancer is a common malignant tumor, and its incidence has been increasing worldwide in recent years. Typical symptoms of endometrial cancer include irregular vaginal bleeding, vaginal discharge, and abdominal pain, and patients at the advanced stage may experience anemia, weight loss, and cachexia [1, 2]. Endometrial carcinoma has been classified into Type I and Type II. Type I, i.e., endometrioid type, because it is similar to the endometrium and is characterized by genetic predisposition, such as obesity, polycystic ovarian syndrome, anovulatory cycles, and irregular menstruation that causes a hyperestrogenic state. Type II cancers are associated with higher patient age, higher stage and grade, nonendometrioid histology, and poor prognosis instead. Most patients with endometrial cancer have an excess of estrogen and typically show a clinical profile of high body mass index, often with other components of metabolic syndrome. Common complications of endometrial cancer include endometrial polyps, breast cancer, uterine fibroids, and ovarian tumors [3]. Laparoscopy is a fiberoptic light source endoscope used for intraabdominal examination and treatment of endometrial cancer. Laparoscopy is completely painless and allows a clear view of the patient's abdominal cavity to understand the cause of the disease [4–6]. A scientific approach in the management of care, using incentives to adequately meet the needs of patients, can fully motivate patients for treatment. Motivation is the process of psychological activities that motivate people through external stimuli to progress towards the desired goal. Motivation in nursing boosts patient motivation in therapy [7–10]. ESCA, according to the definition by Orem, is one's learned capability to engage in self-care behaviors. It has been reported that a good self-care agency predicts favorable adherence to medications, well-preserved quality of life, and a low rate of complications. There are few studies on the improvement of patients' physical and mental health and living conditions after laparoscopic hysterectomy, especially from the perspective of ESCA. To this end, this study examined the rehabilitation effect of incentive nursing on patients with endometrial cancer after laparoscopic hysterectomy to provide a reference for future clinical practice.

## 2. Materials and Methods

### 2.1. General Information

A total of 110 patients with endometrial cancer receiving laparoscopic hysterectomy in our hospital from October 2017 to July 2020 were recruited and randomly assigned (1 : 1) to receive either routine nursing (control group) or incentive nursing plus routine care (study group). The patients in the control group were aged 41–65 years, and those in the study group were aged 42–65 years. The research was approved by the Ethics Committee of our hospital.

### 2.2. Inclusion and Exclusion Criteria

Inclusion criteria were as follows: all patients diagnosed with endometrial cancer received treatment in our hospital; with complete clinical data; with consent to the experiment; aged 30–65 years; with no other serious organ diseases; and provided written informed consent. Exclusion criteria were as follows: patients with death, physical disability, pregnancy, or other autoimmune diseases; with other chronic diseases, hospital referral, mental illness, language dysfunction, or other diseases that affect the results of this study during treatment.

### 2.3. Methods

Surgical methods: Laparoscopic hysterectomy was performed in both groups. With the patient in a lithotomy position, the patient was given anesthesia, followed by the placement of a uterine manipulator through the vagina, and pneumoperitoneum was constructed using carbon dioxide. Laparoscopic exploration was performed with intraabdominal pressure maintained within 14 mmHg. An incision of about 5 mm was made on the left and right lower abdomen as the second and third puncture ports, and a 5 mm incision was made between the symphysis pubis and the umbilical cord as the fourth puncture port. The abdominal cavity and pelvic cavity conditions of the patient were explored, and enlarged and suspicious lymph nodes were removed. Extrafascial hysterectomy and double adnexectomy were performed for the relevant lesions that invaded the myometrium <50%, with a diameter of less than 2 cm, moderately or highly differentiated, and low-risk lymph node metastasis. For lesions with high-risk factors that invade ≥50% of the muscularis, in addition to pelvic lymph node resection, para-aortic lymph nodes were also removed. For lesions involving the cervix, radical hysterectomy was performed, and the abdomen was routinely sutured after lymph node dissection.

#### 2.3.1. Nursing Method

The control group was given routine nursing. Diet nursing: The patients were given health education by the nursing staff, and a diet plan with low sugar, low fat, moderate protein, high fiber, and high vitamins was developed for the patients. Proper exercise: Proper exercise could enhance the body's immunity and improve postoperative recovery. Patients were instructed to participate in appropriate aerobic exercises such as jogging and yoga.

The study group received incentive nursing based on the control group. Health education: The patients were given disease knowledge education, such as common treatments and adverse effects of endometrial cancer, daily dietary guidance, and lifestyle. The patients and their families were lectured by the nurses about endometrial cancer and given incentive psychological counseling to encourage patients to actively participate in the care and treatment in order to improve their self-care ability and self-psychological ability. A medical file was established for the patient, and a care plan was developed according to the patient's condition. Endometrial cancer specialists were invited to lecture patients weekly about exercise, diet, and disease-related knowledge. Telephone follow-up was conducted weekly, and the patient's data were collected and analyzed. Questionnaires were distributed and collected by professional nursing staff at admission and 1 month after discharge. Psychological nursing: The nurse patiently cooperated with the family to care for, support, and encourage the patient. Psychological care was provided according to the patient's personality and psychological characteristics to eliminate their psychological stress and help the patient better cope with various psychological problems in disease treatment. For patients with excessive stress and mood swings during hospitalization, nurses should give psychological counseling and motivation to encourage the patient's cooperation with treatment.

The two groups of patients were given pain care. After surgical treatment, a long healing time of the wound may lead to local pain. The patients were given analgesic injections as prescribed for pain relief within 6–24 h postoperatively. An intramuscular injection of pertechnetate hydrochloride 50–90 mg was administered with a controlled frequency of 2–3 injections. For patients with stronger postoperative pain, analgesic pumps were used to reduce the risk of pulmonary infections, and nursing interventions such as turning, deep breathing, and coughing up sputum were provided. Infection prevention: Patients with endometrial cancer were prone to different degrees of infection after surgery, which compromised their recovery. Therefore, postoperative vital signs of the patients were monitored continuously for 1 week by nursing staff, and the patients were instructed to drink more water, urinate more, and exercise appropriately to reduce the risk of infection from their surgical incisions. For patients with abdominal drains indwelling after surgery, nursing staff should enhance laboratory tests regarding the flow, the color, and properties of the patient's urine while avoiding pressure and distortion of the urinary catheter and changing the drainage bag regularly.

### 2.4. Outcome Measures

1. Self-rating anxiety scale (SAS) [11] score was used to evaluate the patients' anxiety with a total score of 100 points. A score of 50–70 points indicates mild anxiety, a score of 71–90 points indicates moderate anxiety, and a score of >90 points indicates severe anxiety.
2. Hamilton depression scale (HAMD) [11] was used to evaluate the depression of patients. The scale includes 24 items, and the higher the score, the more serious the depression.
3. The exercise of self-care agency (ESCA) was used to evaluate the self-care ability with a confidence validity of 0.865. The ESCA was divided into 4 dimensions (self-care concept, self-care responsibility, self-care skills, and health knowledge level), with 43 items and a total score of 172 points. The higher the score, the stronger the self-care ability.
4. Rehabilitation: The time of the first postoperative out-of-bed activities, the time of the first exercise, and the length of hospital stay in the two groups were recorded and compared.
5. Complications: Complications that may occur during postoperative care include fever, irregular vaginal bleeding, abdominal pain, and uterine infection. The equation for incidence of complication is the number of complications divided by the total number of participants.
6. Nursing Satisfaction: The Nursing Satisfaction Questionnaire made by our hospital was used, with a total of 20 questions, with 5 points for each question. A total score of <70 points indicates unsatisfied, a score of 70–89 points indicates satisfied, and a total score of ≥90 points indicates highly satisfied. Satisfaction = (highly satisfied cases + satisfied cases)/Total cases × 100%.

### 2.5. Statistical Methods

SPSS20.0 was used for data analysis, and GraphPad Prism 8 was used to plot the graphs. Measurement data were expressed as ($\bar{\text{x}}$ ±*s*) and processed by the independent sample t-test. The counting data were expressed as the number of cases (rate) and processed by the *X*^2^ test. Differences were considered statistically significant at *P* < 0.05.

## 3. Results

### 3.1. Baseline Data

There was no significant difference in the general data such as age, body weight, stage of endometrial cancer, and type of endometrial cancer between the two groups (*P* > 0.05). (Table 1).

### 3.2. SAS Score

The two groups showed similar SAS scores before treatment (82.21 ± 5.14 vs. 82.17 ± 5.09) (*P* > 0.05). Patients receiving incentive nursing showed significantly lower SAS scores (42.34 ± 3.85) versus patients given routine care alone (71.15 ± 4.32) (*P* < 0.05) (Table 1). (^*∗*^indicates a significant difference in the comparison of SAS scores between the control group and the study group before nursing, *t* = 0.041, *P*=0.967) (^*∗∗*^indicates a significant difference in the comparison of the SAS scores between the control group and the study group after nursing, *t* = 36.923, *P* < 0.001) (Figure 1).

### 3.3. HAMD Score

There was no statistical significance in the HAMD score between the two groups before treatment (65.82 ± 4.28 vs. 65.91 ± 4.11) (*P* > 0.05). Incentive care was associated with a significantly lower HAMD score (41.38 ± 3.46) versus routine nursing (55.12 ± 3.56) (*P* < 0.05) (Figure 2). (^*∗*^indicates a significant difference in the comparison of HAMD scores between the control group and the research group before nursing treatment, *t* = -0.112, *P*=0.911) (^*∗∗*^indicates a significant difference in the comparison of the HAMD scores between the control group and the research group after nursing treatment, *t* = 20.526, *P* < 0.001).

### 3.4. ESCA Score

The two groups showed comparable ESCA scores before treatment (*P* > 0.05). Incentive care was associated with a significantly higher ESCA score versus routine nursing (*P* < 0.05). (Table 2).

### 3.5. Postoperative Rehabilitation

Incentive care resulted in a shorter length of hospital stay (10.85 ± 4.21) d and postoperative time to out-of-bed activities (4.67 ± 2.12) d and exercises (7.31 ± 2.03) d versus routine care ([8.63 ± 3.45] d, [3.12 ± 1.76], and [5.27 ± 2.12]) (*P* < 0.05). (Table 3).

### 3.6. Comparison of the Incidence of Complications in Patient Care

Incentive care was associated with a significantly lower incidence of nursing complications (4%, including 1 case of fever and 1 case of intrauterine) versus routine nursing (16%, including 3 cases of fever, 1 case of irregular vaginal bleeding, 3 cases of abdominal pain, and 2 cases of intrauterine infection) (*P* < 0.05). (Table 4).

### 3.7. Nursing Satisfaction

Incentive care resulted in significantly higher nursing satisfaction (94%, including 33 cases of highly satisfied, 19 cases of satisfied, and 3 cases of dissatisfied) versus routine nursing (67%, including 27 cases of highly satisfied, 10 cases of satisfied, and 18 cases of dissatisfied) (*P* < 0.05). (Table 5).

## 4. Discussion

Endometrial cancer is an epithelial malignant tumor that occurs in the endometrium of women, to which perimenopausal and postmenopausal women are more susceptible. It can be divided into endometrioid adenocarcinoma, adenocarcinoma with squamous cell differentiation, and mucinous adenocarcinoma. In recent years, its incidence has been increasing worldwide [11–14]. Compared with laparotomy, laparoscopic surgery is less traumatic with less intraoperative blood loss, which contributes to the postoperative recovery of patients. Laparoscopy allows for a more open view of the organization of anatomical structures, which facilitates the exposure of blood vessels deep in the occluded fossa, clearly excises the lymph nodes in the area, and avoids extensive damage to blood vessels deep in the occluded fossa. In addition, the construction of the pneumoperitoneum can effectively increase abdominal pressure and avoid damage to small blood vessels [15–18]. Accordingly, laparoscopic surgery was adopted in the present study. Moreover, incentive nursing was also used to mobilize the patients for better treatment and nursing cooperation [19–21]. Negative emotions such as fear and anxiety lead to a significant weakening of the body's “immune surveillance” (which is often regarded as the intellectual underpinning of cancer immunology). Although the hypothesis itself has contributed little to our attempts to treat cancer through immunological means, it has profound implications for understanding the functions of the immune system., “while a good psychological condition can promote the body's recovery”. To alleviate and eliminate the patient's negative emotions and enhance the immunity of the organism, the nursing staff should give priority to the patient's health and recovery and provide the patient with as much attentive service as possible.

In the present study, patients receiving incentive nursing showed significantly lower SAS scores and HAMD scores versus patients given routine care alone, indicating that incentive nursing is effective in reducing anxiety and depression. Studies have shown that anxiety disorders are associated with poor recovery outcomes and increased medical complications in patients with endometrial cancer, compromising their quality of life. The study group outperformed the control group in terms of ESCA scores, which indicated that incentive nursing can effectively improve the self-management ability of patients. Furthermore, incentive care herein resulted in a shorter length of hospital stay and postoperative time for out-of-bed activities and exercises versus routine care, which indicates that incentive nursing can boost postoperative recovery. Also, incentive care was associated with a significantly lower incidence of nursing complications versus routine nursing, suggesting that incentive nursing can enhance the patients' understanding of the disease, which results in better protection and reduces the incidence of nursing complications.The results of nursing satisfaction showed a higher satisfaction was found in patients given incentive nursing versus routine nursing, which further proved the feasibility of incentive nursing. Comprehensive care of endometrial cancer patients using the holistic concept of traditional Chinese medicine, including care of the patient's physique, personality, mood, and dietary habits, as well as attention to the effects of climate and geography, can achieve promising nursing outcomes. All these findings are attributed to the fact that incentive nursing is implemented throughout the whole process by motivating the patients and their family members in various aspects. Conversely, the traditional one fails to focus on these but considers them a matter of routine instead.

Moreover, previous studies suggested that DNA methylation inhibitors were administered to endometrial cancer cell lines to determine their ability to inhibit cell growth and analyze the downstream genes regulated by DNA methylation. Histone deacetylase (HDAC) inhibitors have been reported to induce apoptosis in endometrial cancer cell lines. Several studies have investigated the combination of HDAC inhibitors and other anticancer agents, such as carboplatin, docetaxel, gemcitabine, cisplatin, etoposide, doxorubicin, and paclitaxel in gynecological cancers. HDAC inhibitors have also been reported to restore the expression of progesterone receptors in endometrial cancer cells. Moreover, it was proven that HDAC inhibitors suppressed the oncogene MYC in EC cells. Vorinostat is also effective in endometrial cancer cell lines. It is considered that the insulin-like growth factor system is related to the carcinogenesis of endometrial cancer and that vorinostat was found to induce apoptosis by suppressing its insulin-like growth factor signals [22–24].

## 5. Conclusion

Incentive nursing can effectively improve the ESCA level of patients, promote postoperative recovery, and reduce the incidence of complications, so it is worthy of clinical promotion.

## Figures and Tables

**Figure 1:** Comparison of SAS scores before and after nursing treatment (*x* ± *s*).

**Figure 2:** Comparison of HAMD scores before and after nursing treatment (*x* ± *s*).

**Table 1:** Comparison of general data of the two groups of patients (*n* (%)).

	Control group (*n* = 55)	Study group (*n* = 55)	*T* Or *x*^2^	*P*
Average age (years)	55.21 ± 3.35	55.30 ± 3.24	−0.143	0.887
Average weight (kg)	60.12 ± 8.02	60.33 ± 7.98	−0.138	0.89
Endometrial cancer staging			0.178	0.673
Stage I	39	37		
Stage II	15	17		
Stage III	1	1		
Stage IV	0	0		
Endometrial cancer typing			0.178	0.673
Endometrioid adenocarcinoma	39	37		
Adenocarcinoma with squamous cell differentiation	15	17		
Clear cell carcinoma	1	1		

**Table 2:** Comparison of ESCA scores before and after nursing treatment (*x* ± *s*).

Group	Cases	ESCA							
		Self-care concept		Self-care responsibility		Self-care skills		Health knowledge level	
		Before treatment	After treatment	Before treatment	After treatment	Before treatment	After treatment	Before treatment	After treatment
Control group	55	20.11 ± 5.02	25.31 ± 3.14	20.36 ± 4.42	24.38 ± 6.10	30.14 ± 3.32	34.22 ± 3.97	33.24 ± 7.05	40.12 ± 4.31
Study group	55	20.08 ± 4.99	30.17 ± 3.44	20.33 ± 4.38	31.49 ± 7.21	30.11 ± 3.27	43.21 ± 4.18	33.25 ± 7.08	47.52 ± 4.66
t	—	0.031	−7.738	0.036	−5.583	0.048	−1.565	−0.007	−8.646
P	—	0.975	<0.001	0.971	<0.001	0.962	<0.001	0.994	<0.001

**Table 3:** Comparison of postoperative rehabilitation progress of patients (*x* ± *s*).

Group	Cases	Postoperative recovery process of patients		
		The first time to get out-of-bed after surgery (d)	The first time to participate in sports after surgery (d)	Hospital stay (d)
Control group	55	4.67 ± 2.12	7.31 ± 2.03	10.85 ± 4.21
Study group	55	3.12 ± 1.76	5.27 ± 2.12	8.63 ± 3.45
T	—	4.172	5.154	3.025
P	—	<0.001	<0.001	0.003

**Table 4:** Comparison of complication rates among patients (*n* (%)).

Group	Cases	Fever	Irregular vaginal bleeding	Bellyache	Intrauterine infection	Total incidence
Control group	55	3	1	3	2	9 (16%)
Study group	55	1	0	0	1	2 (4%)
x^2^	—	—	-	-	-	4.949
P	—	—	-	-	-	0.026

**Table 5:** Comparison of patient care satisfaction (*n* (%)).

Group	Cases	Great satisfaction	Satisfaction	Dissatisfaction	Total satisfaction
Control group	55	27	10	18	37 (67%)
Study group	55	33	19	3	52 (94%)
*x* ^2^	—	—	—	—	13.242
P	—	—	—	—	<0.01

## Data Availability

The datasets used during the present study are available from the corresponding author upon reasonable request.
